The article "IoT-Oriented 6G Wireless Network System for Smart Cities" was published in 2022. Journal: Comput Intell Neurosci.

# IoT-Oriented 6G Wireless Network System for Smart Cities

**DOI:** 10.1155/2022/1874436

**Published:** 2022-08-10

**Authors:** M. M. Kamruzzaman, Md Altab Hossin, Omar Alruwaili, Saad Alanazi, Madallah Alruwaili, Nasser Alshammari, Alaa Alaerjan, Roksana Zaman

**Affiliations:** ^1^Department of Computer Science, College of Computer and Information Sciences, Jouf University, Sakakah, Saudi Arabia; ^2^School of Innovation and Entrepreneurship, Chengdu University, No. 2025 Chengluo Avenue, Chengdu 610106, Sichuan, China; ^3^Department of Computer Engineering and Networks, College of Computer and Information Sciences, Jouf University, Sakakah, Saudi Arabia; ^4^School of Electrical and Information Engineering, Tianjin University, Tianjin, China

## Abstract

The smart city is an emerging concept that is based on the integration of various electronic devices and citizens that enhance the flow of information. IoT is an integral part for next generation wireless network infrastructure for acting as an interface of collecting data and controlling delivery of message which are using in smart cities. In this paper, an IoT-oriented relay assisted MIMO for beyond the fifth-generation wireless network system is proposed. The proposed system provides higher capacity and lower BER. The proposed system's BER results are compared with various combinations of transmission and receiving antennas at source, relay, and destination. It is found from BER performance that the developed scheme with relay does provide 1–17 dB gain with respect to direct connection. It is also found from mathematical analysis and simulation results that this scheme provides 3 to 9 b/s/Hz improvement in performance of capacity at 5 to 10 dB by adding a different combination of STBC and VBLAST. Simulation results are also presented to demonstrate the diversity and multiplexing gain that is a key to providing high data rates with reliable communication with many interferences for the IoT system. This system can also be used for massive antennas-based IoT system by raising the number of transmitting and receiving antennas with proposed encoding and decoding techniques explained in this paper.

## 1. Introduction

The smart city is an emerging concept that is based on the integration of various electronic devices and citizens that enhance the flow of information. Smart city is the city that has an intelligent, integrated, and cost-effective technology that connects different aspects of the cities such as transportation, resource usage, waste management, and human health. These systems are critical in handling the challenges caused by the massive urbanization of cities that have led to population increase along with issues such as traffic congestion, poor health management, and environmental unsustainability. Thus, smart cities can play a massive role in the improvement of the lives and health of the citizens through advanced management.

The article "IoT-Oriented 6G Wireless Network System for Smart Cities" was published in 2022. Journal: Comput Intell Neurosci.

Wireless communication for the next-generation, such as 5G and beyond, is considered to be extremely dynamic and complex. The advancement of ultradense heterogeneous network deployment, high capacity and low BER, and new applications necessitate a new framework for wireless communication that may pose numerous critical challenges of network operation, management, planning, designing, and troubleshooting. At the same time, the generation and consumption of wireless data is shifting from people-centric to machine-oriented communications, making future wireless network operations even more complex. As a result, new methodologies for employing distributed computational means with better context perception will become increasingly important in order to reduce the complexity of future wireless network operations.

6G will be transformative and will revolutionize the wireless evolution with more stringent requirements such as higher capacity, lower latency, extensive connectivity, higher security, high quality of experience, low consumption of energy, and stable connection which can be used in smart cities. Wireless communication system is considered as one of the most important components of Internet of Things (IoT) infrastructure. This element serves as the bridge for dual communication for control message delivery and data gathering. In IoT, a huge number of users' devices with sensors or without sensor are linked and communicate through tactile Internet, and that is the fundamental feature IoT which will allow real-time communication among systems with a range of activities of community, high tech industry, and commercial use [1, 2].

Currently, there are millions of smartphone and smart sensor devices. Number of electronic devices which linked with Internet is increasing exponentially to realize the concept of IoT. Smartphone users annually rising with the rate of approximately 25 percent and it is anticipated that it would reach eighty billion by the end of the year 2030. Therefore, for designing and deploying 6G in IoT, the notion of 6G, its requirements, as well as the required technologies must be thoroughly investigated [3]. A smart city employs all new network technologies, such as 6G, cloud, mobile Internet, IoT, edge, fog computing, and so on, to create a cost-effective and efficient interaction with all IoT devices in the city [4].

IoT-oriented wireless network will face various challenges for managing the large aspects in heterogeneous traffic including meeting all service-quality criteria such as monitoring network reliability, maintaining data security, achieving a cost-effective way for an efficient network deployment, exploration with a focus on distant and stand-alone locations, lowering the cost of wireless communications use, increasing the longevity of battery life of mobile devices, and the achievement of a maximum data rate. In order to handle those challenges and develop a generalized 6G infrastructure, architectural requirements, supporting technologies, and related security threats and countermeasures should be analyzed firstly. The deployment of 6G in IoT is expected to generate different forms types of traffic, energy consumption, bit rates, reliability, and privacy, and security. The main objective behind this work is to address the IoT-oriented 6G cellular network to meet the data needs that are expected by increasing with the deployment of a massive number of devices.

The article "IoT-Oriented 6G Wireless Network System for Smart Cities" was published in 2022. Journal: Comput Intell Neurosci.

There are primarily two schemes for deploying multiple antennas at the relay. The first is transmit diversity, which involves sending multiple copies of the same transmission sequence through different transmission antennas. Space Time Block Coding (STBC) is a common transmit diversity approach. The other is spatial multiplexing, which involves sending different transmission sequences through various transmission antennas. Vertical Bell Labs Layered Space Time (VBLAST) is a common transmitting multiplexing approach. However, STBC has a lower spectral efficiency than VBLAST because it does not provide multiplexing gain. VBLAST, on the other hand, has the drawbacks of having a higher BER than STBC because it does not provide the diversity gain.

The present research proposes relay assisted IoT-oriented wireless network system using Multiple Input Multiple Output (MIMO) technique. There are several research studies on MIMO for IoT; such as, Massive MIMO connectivity for the Internet of Things (IoT) is studied to recognize the benefits and challenges of using massive MIMO with IoT [5–7]. Overlapping among grouping for users is investigated for IoT-related massive MIMO wireless network systems [8]. A multilayer and hybrid MIMO system for wireless communication is studied in [9–11]. A novel design approach for 5G Massive MIMO and NB-IoT green networks using a hybrid Jaya-differential evolution algorithm is proposed [12]. Reference [13] shows zero-forcing-based downlink virtual MIMO–NOMA communications in IoT networks. Reference [14] proposes a new leakage-based precoding scheme in IoT-oriented cognitive MIMO-OFDM Systems. As per the researcher's knowledge, relay assisted IoT-oriented wireless network studies are unprecedented in the previous literature [15–17]. Nevertheless, the suggested relay assisted IoT-oriented MIMO using combination of STBC and VBLAST scheme attains better multiplexing gain and diversity, while providing high capacity and low BER that assist in sustaining system's reliability. The proposed system can also be used for massive antennas-based IoT system raising the number of transmitting and receiving antennas with proposed encoding and decoding techniques explained in this paper. Massive MIMO is a key enabling technology for next-generation mobile communication that combines antennas at both the transmitter and the receiver to have higher spectral and energy efficiency with relatively simple technique. Due to the shortage of bandwidth world-wide in the mobile communication, industry has prompted the research and exploration of massive MIMO.

The article "IoT-Oriented 6G Wireless Network System for Smart Cities" was published in 2022. Journal: Comput Intell Neurosci.

The remainder of this paper is organized as follows. Section 2 describes the system model where it explains sensor layer, IoT gateway, encoding, and decoding techniques at relay and base station. This section also shows the analysis of BER, capacity, diversity, and multiplexing gain. Finally, Section 3 concludes the paper with the direction of future work.

## 2. System Model

Figure 1 shows the IoT-oriented 6G framework which shows applications where smart sensors are used, sensor layers, IoT gateway, and relay and base station. Following section are explained in detail:

### 2.1. Sensor Layer

The layer incorporates smart sensor-based devices such as smart home having temperature control, air conditioners, refrigerator, fan, and light. It is important to note that smart sensors are a combination of interfacing units and sensors. These sensors have the capability of conducting 2-way communication while supporting decision making and communication activities. In IoT, this layer carries out a machine type communication (MTC), while communicating with gateway.

### 2.2. IoT Gateway

This layer is utilized for providing long-range and low power connectivity to the IoT applications.

In this account, there is a possibility of multiple connections for achieving critical and massive IoT connectivity via low power wide area networks (LPWANs). The rationale behind using LPWA technology in IoT application is that they possess unique characteristics, particularly, high data rates, better energy efficiency, low power consumption, and wide-area coverage.

### 2.3. Relay and Base Station

Relay and Base station belong to the communication layer which is regarded to be the IoT architecture's backbone because it is responsible for transferring all the information in the layers. Besides, various technologies including radio frequencies, mm-wave radio frequencies, and coding and massive MIMO are considered in this layer.

The article "IoT-Oriented 6G Wireless Network System for Smart Cities" was published in 2022. Journal: Comput Intell Neurosci.

An uplink wireless communication is taken into consideration for evaluating the performance. Here, two to eight antennas (*M*_*T*_=2 to 8) are allotted in the proposed system which can be extended for massive MIMO system using same encoding technique. Besides, the relay has *M*_*R*_ and *N*_*R*_ transmitting and receiving antennas, respectively. As depicted in Figure 2, the destination has *N*_*B*_ receiving antenna. For encoding information at source, an STBC encoder is utilized. However, for re-encoding information at the relay, MLSTBC is utilized. The detailed explanation of the encoding with the help of STBC, re-encoding and decoding with the help of combined STBC-VBLAST at the relay, and decoding via ML at the destination is provided in the proceeding sections.

#### 2.3.1. Encoding at Source

The bit sequences of the information, i.e., *b*_k_ is moderated by a modulator such as 64 QAM or 16 QAM or QPSK. However, the encoding of the modulated symbols is conducted by STBC; here, *k* denotes the number of sources. On the other hand, the encoded system is represented by *x*_*k*,*i*,*t*,*j*_. Here,

*i* signifies the symbol number.

*j* is transmit antenna *M*_*T*_.

*t* is time slot.

Table 1 shows the encoding at source for transmitting from two transmission antennas using encoding technique of STBC. The transmitted signal of the first antenna at the first time slot of the kth user is signified by *x*_*k*,1,1,1_ and from the second antenna by *x*_*k*,2,1,2_. Likewise, in the second time slot, the signals −*x*_*k*,2,2,1_^*∗*^ and *x*_*k*,1,2,1_^*∗*^ are transmitted from the first and second antennas, respectively. Here, ^*∗*^signifies the operation of complex conjugate.

#### 2.3.2. Decoding the Signal Received at Relay

Symbols' vectors—that are obtained from source (i.e., STBC transmitters) during t*1* (first time slot) can be shown as

(1) $$\begin{array}{c} R_{t1}=\sqrt{\frac{E_{x}}{KM_{T}N_{0}}}U_{\text{STBC}}^{t1}X_{\text{STBC}}+N_{t1}. \end{array}$$

Here,

(2) $$\begin{array}{c} R_{t1}=\left[\begin{array}{c} \begin{array}{c} r_{1}^{1}\\ r_{2}^{1} \end{array}\\ \begin{array}{c} \vdots \\ r_{N_{R}}^{1} \end{array} \end{array}\right],\\ U_{STBC}^{t1}=\left[\begin{array}{ccccccc} u_{1_{11}} & u_{1_{12}} & u_{2_{11}} & u_{2_{12}} & \ldots & u_{K_{11}} & u_{K_{12}}\\ u_{1_{21}} & u_{1_{22}} & u_{2_{21}} & u_{2_{22}} & \ldots & u_{K_{21}} & u_{K_{22}}\\ \vdots & \vdots & \vdots & \vdots & \ddots & \vdots & \vdots \\ u_{1_{N_{R}1}} & u_{1_{N_{R}2}} & u_{2_{N_{R}1}} & u_{2_{N_{R}2}} & \ldots & u_{K_{N_{R}1}} & u_{K_{N_{R}2}} \end{array}\right],\\ l=1,\ldots ,N_{R},\\ X_{STBC}=\left[\begin{array}{c} x_{1,1}\\ x_{1,2}\\ x_{2,1}\\ \begin{array}{c} x_{2,2}\\ \begin{array}{c} \vdots \\ x_{K-1,1}\\ x_{K,2} \end{array} \end{array} \end{array}\right],\\ N^{t1}=\left[\begin{array}{c} \begin{array}{c} n_{1}^{1}\\ n_{2}^{1} \end{array}\\ \begin{array}{c} \vdots \\ n_{N_{R}}^{1} \end{array} \end{array}\right]. \end{array}$$

However, the signal received at t*2* (second time slot) at relay can be shown as

(3) $$\begin{array}{c} R^{t2}=\sqrt{\frac{E_{x}}{KM_{T}N_{0}}}U_{\text{STBC}}^{t2}X_{\text{STBC}}+N_{t2}. \end{array}$$

Here,

(4) $$\begin{array}{c} R^{t2}=\left[\begin{array}{c} \begin{array}{c} r_{1}^{2*}\\ r_{2}^{2*} \end{array}\\ \begin{array}{c} \vdots \\ r_{N_{R}}^{2*}\;\;\; \end{array} \end{array}\right],\\ U_{\text{STBC}}^{t2}=\left[\begin{array}{ccccccc} u_{112}^{*} & -u_{111}^{*} & u_{212}^{*} & -u_{211}^{*} & \ldots & u_{K12}^{*} & -u_{K11}^{*}\\ u_{122}^{*} & -u_{121}^{*} & u_{222}^{*} & -u_{221}^{*} & \ldots & u_{K22}^{*} & -u_{K21}^{*}\\ \vdots & \vdots & \vdots & \vdots & \ddots & \vdots & \vdots \\ u_{1N_{R}2}^{*} & -u_{1N_{R}1}^{*} & u_{2N_{R}2}^{*} & -u_{2N_{R}1}^{*} & \ldots & u_{KN_{R}2}^{*} & -u_{KN_{R}1}^{*} \end{array}\right],\\ N^{t2}=\left[\;\;\;\;\begin{array}{c} \begin{array}{c} n_{1}^{2*}\\ n_{2}^{2*} \end{array}\\ \begin{array}{c} \vdots \\ n_{N_{R}}^{2*}\;\;\; \end{array} \end{array}\right]. \end{array}$$

The combination of the received signal *R*_STBC_ for *t1* and *t2* is represented as

(5) $$\begin{array}{c} R_{\text{STBC}}=U_{\text{STBC}}X_{\text{STBC}}+N_{\text{STBC}}. \end{array}$$

Here,

(6) R=STBCRt1Rt2,U=STBCUSTBCt1USTBCt2,N=STBCNt1Nt2.

The article "IoT-Oriented 6G Wireless Network System for Smart Cities" was published in 2022. Journal: Comput Intell Neurosci.

The transmitted signal can be estimated by ${\hat{R}}_{\text{STBC}}$ as shown below:

(7) $$\begin{array}{c} {\tilde{R}}_{\text{STBC}}=U_{\text{STBC}}^{H}R_{\text{STBC}},\\ =\sqrt{\frac{E_{x}}{KM_{T}N_{0}}}U_{\text{STBC}}^{H}U_{\text{STBC}}X_{\text{STBC}}+U_{\text{STBC}}^{H}N_{\text{STBC}},\\ =\sqrt{\frac{E_{x}}{KM_{T}N_{0}}}U_{STBC}X_{\text{STBC}}+U_{\text{STBC}}^{H}+{\tilde{N}}_{\text{STBC}}. \end{array}$$

Following ML technique is used to detect the symbol from (3):

(8) $$\begin{array}{c} {\tilde{x}}_{i,ML}=Q\left(\frac{{\tilde{R}}_{\text{STBC},i}}{\sqrt{\left(E_{x}/KM_{T}N_{0}\right)}U_{\text{STBC}}^{H}U_{\text{STBC}}}\right),\\ i=1,2,\ldots ,2K. \end{array}$$

Here, Slicing function Q(.) is used to find a symbol transmitted from transmit antennas from the respective constellation set.

#### 2.3.3. Re-Encoding by Utilizing Combined STBC-VBLAST at Relay

In the proposed system, the technique of combine STBC-VBLAST is utilized for re-encoding the transmitted information. Besides, the alleged G2 of STBC scheme is also utilized for implementing the system. It is important to note that other STBC schemes can also be used, such as H4, H3, G4, and G3 depending on the network needs [18, 19]. As presented in Table 2, if one VBLAST layer and one STBC groups are utilized, it is represented as G21. However, as depicted in Table 3, if two VBLAST layers and one STBC groups are utilized, it is represented as G211. Likewise, as illustrated in Table 4, if two VBLAST layers and STBC groups are utilized, it is represented as G2G211.

The article "IoT-Oriented 6G Wireless Network System for Smart Cities" was published in 2022. Journal: Comput Intell Neurosci.

Generally, the systems' transmitted signals can be represented in the matrix form as

(9) $$\begin{array}{c} X=\left[\begin{array}{c} \begin{array}{c} x_{1_{\text{VBLAST}}}\\ x_{2_{\text{VBLAST}}}\\ \vdots \\ x_{L_{\text{VBLAST}}} \end{array}\\ \begin{array}{c} x_{1_{\text{STBC}}}\\ x_{2_{\text{STBC}}}\\ \vdots \\ x_{L_{\text{STBC}}} \end{array} \end{array}\right]. \end{array}$$

Here, *x*_*i*_VBLAST__/*x*_*i*_*STBC*__  = Transmitted symbols of *i*^*th*^ VBLAST/STBC layer of combined STBC-VBLAST.

*X* can be rewritten as

(10) $$\begin{array}{c} X=\left[\begin{array}{c} \begin{array}{cc} {\hat{x}}_{1} & -{\hat{x}}_{2}^{*}\\ {\hat{x}}_{3} & -{\hat{x}}_{4}^{*}\\ \vdots & \vdots \\ \vdots & \vdots \\ {\hat{x}}_{n-1} & -{\hat{x}}_{n}^{*} \end{array}\\ \begin{array}{cc} {\hat{x}}_{n+1} & {\hat{x}}_{n+2}\\ -{\hat{x}}_{n+2}^{*} & {\hat{x}}_{n+1}^{*}\\ \vdots & \vdots \\ \vdots & \vdots \\ {\hat{x}}_{n-1} & {\hat{x}}_{n}\\ -{\hat{x}}_{n}^{*} & {\hat{x}}_{n-1}^{*} \end{array} \end{array}\right]. \end{array}$$

#### 2.3.4. Decode Symbols at Destination

The received signal can be shown as follows:

(11) $$\begin{array}{c} r=H\left[\begin{array}{c} \begin{array}{c} x_{1_{\text{VBLAST}}}\\ x_{2_{\text{VBLAST}}}\\ \vdots \\ x_{L_{\text{VBLAST}}} \end{array}\\ \begin{array}{c} x_{1_{\text{STBC}}}\\ x_{2_{\text{STBC}}}\\ \vdots \\ x_{L_{\text{STBC}}} \end{array} \end{array}\right]+n. \end{array}$$

After rearrangement, (6) can be demonstrated as

(12) $$\begin{array}{c} r=H_{\text{combine STBC}-\text{VBLAST}}X_{\text{ combine STBC}-\text{VBLAST}}+n, \end{array}$$

Here, **r**=$\left[\begin{array}{c} r_{1}\\ r_{2}^{*}\\ \vdots \\ r_{{\left(n_{R}\right)}_{D}-1}\\ r_{{\left(n_{R}\right)}_{D}}^{*} \end{array}\right]$ is the received signal, $H_{\text{combine STBC}-\mathrm{VBLAST}}=\left[\begin{array}{cccc} {\text{H}}_{\text{VBLAST}}^{1} & {\text{H}}_{\text{VBLAST}}^{2} & \cdots & {\text{H}}_{\text{VBLAST}}^{\text{l}}\begin{array}{cccc} {\text{H}}_{\text{STBC}}^{1} & {\text{H}}_{\text{STBC}}^{2} & \cdots & {\text{H}}_{\text{STBC}}^{\text{l}} \end{array} \end{array}\right]$

Is the 1 to *l* of STBC and VBLAST group's channels.

**X**_combine STBC−VBLAST_ is the transmitted symbols transmitting in *t*1 and *t*2. However, **n**=$\left[\begin{array}{c} n_{1}\\ n_{2}^{*}\\ \vdots \\ n_{{\left(n_{R}\right)}_{D}-1}\\ n_{{\left(n_{R}\right)}_{D}}^{*} \end{array}\right]$ is regarded to be the noise that is produced at the destination.

$\tilde{r},$ can be used for detecting the transmitting symbols. $\tilde{r},$ is the combination of signals, transmitted from t1 and t2, and can be represented as

(13) $$\begin{array}{c} \tilde{r}=H_{\text{combine STBC}-\text{VBLAST}}^{H}r,\\ \tilde{r}=H_{\text{combine STBC}-\text{VBLAST}}^{H}H_{\text{combine}\text{STBC}-\text{VBLAST}}X+\tilde{n}. \end{array}$$

Detection technique from (14) can be utilized for finding the transmitted symbols. In the proposed system, the ML detector has been utilized for detecting the symbols. Besides, 64 QAM or 16 QAM, or QPSK demodulator are utilized for demodulating the detecting systems and getting the output.

The article "IoT-Oriented 6G Wireless Network System for Smart Cities" was published in 2022. Journal: Comput Intell Neurosci.

#### 2.3.5. Analysis of BER

There is a chance that errors will be created into the system when information is transmitted across a transmission link. If errors are initiated into the information, the system's consistency may be adversely affected. As a result, it is necessary to examine the performance of a system, and bit error rate, or BER, is an ideal method for doing so. Unlike all the other types of evaluation, BER evaluates the entire end-to-end system performance, including the sender, receiver, and a medium between sender and receiver. Therefore, BER shows the real performance of a system in operation, instead of evaluating the component parts.

Computer simulation is conducted in this section for showing the proposed system's BER. In this account, the evaluation of the results has been carried out for a different combination of Rx and Tx. For simulations, QPSK has been used. However, it has been assumed that the relay is positioned in the mid of the destination and source.

Proposed system's BER performance for source with 8 antennas is shown in Figure 3. It has been found that the VRL gives gain of 18 dB with comparison of DL at 10^−5^. Likewise, the gain of 12 dB is given by VRL for the different configuration as compared to DL at 10^−5^ for source with 8 antennas.

It has also been found that at low SNR, the performance of G21 is far better as compared to G2G211. Contrarily, G2G211 had shown better performance from 3 dB onward. However, it is established that G211 had shown the worst performance among G2G211, G211, and G21. Therefore, it can be deduced that the addition of VBLAST layer in combined STBC-VBLAST brings negative impacts on the BER performance. On the other hand, the addition of the G2 layer results in improving BER performance for the proposed system.

The article "IoT-Oriented 6G Wireless Network System for Smart Cities" was published in 2022. Journal: Comput Intell Neurosci.

#### 2.3.6. Analysis of Capacity

MIMO with combined STBC-VBLAST system's capacity can be represented as:

(14) $$\begin{array}{c} C_{\text{combine STBC}-\text{VBLAST}}={\text{log}}_{2}\det\left(I_{n_{R}}+\frac{P_{T}}{n_{T}\sigma_{\text{n}}^{2}}H_{\text{combine STBC}-\text{VBLAST}}H_{\text{combine STBC}-\text{VBLAST}}^{H}\right). \end{array}$$

Since combined STBC-VBLAST consists of several STBC blocks and VBLAST layers, we can simplify*H*_combine STBC−VBLAST_ and write (21) as Here, *L*_STBC_  = Number of STBC blocks.*L*_VBLAST_  = Number of VBLAST blocks.

In combined STBC-VBLAST technique, VBLAST layer sends the first symbol at the first time slot and the negative conjugate of the second symbol sends at the second time slot. On the other hand, G2 of STBC was used to send information from STBC block in combined STBC-VBLAST. So, (10) can be further simplified as (11):

(15) $$\begin{array}{c} C_{\text{combine STBC}-\text{VBLAST}}={\text{log}}_{2}\left[\det\left(I_{n_{R}}+\frac{P_{\text{T}}}{n_{T}\sigma_{\text{n}}^{2}}\left(\sum_{i=1}^{L_{\text{VBLAST}}}H_{\text{VBLASTiF}}^{2}+\sum_{j=1}^{L_{\text{STBC}}}H_{\text{STBCjF}}^{2}\right)\right)\right]. \end{array}$$

Proposed system's capacity is shown in Figure 4 for representing the performance of G2G2111, G2G211, G211, and G21.


(16) $$\begin{array}{c} C_{\text{combine STBC}-\text{VBLAST}}={\text{log}}_{2}\det\left(I_{n_{R}}+\frac{{\text{P}}_{T}}{n_{T}\sigma_{\text{n}}^{2}}\left(\sum_{i=1}^{L_{\text{VBLAST}}}H_{{\text{VBLAST}}_{\text{i}}}H_{{\text{VBLAST}}_{\text{i}}}^{H}+\sum_{j=1}^{L_{\text{STBC}}}H_{{\text{STBC}}_{\text{j}}}H_{{\text{STBC}}_{\text{j}}}^{H}\right)\right). \end{array}$$

#### 2.3.7. Analysis of Diversity and Multiplexing Gain

*Diversity Gain*. (*d*). Diversity gain is considered as the measurement of reliability. It represents how swiftly the error probability decays with the increased signal-to-noise ratio (SNR). If a system possesses *n*_*R*_ receiving antennas and *n*_*T*_  transmitting antennas, *n*_*T*_*n*_*R*_ will be achieved as a maximal diversity gain. In a space-time coding scheme, when the maximal diversity gain of *d*_max_ is present, the average error probability *p*_*e*_) can decay as 1/SNR^*d*_max_^. Therefore, diversity gain can be

achieved by a space-time coding scheme, if

(17) $$\begin{array}{c} p_{e}\left(\text{SNR}\right)∼{\text{SNR}}^{-d_{\text{max}}}. \end{array}$$

for a fixed rate of data.

*Degree of Freedom and Spatial Multiplexing Gain* : signals arrive in multiple directions which provide multiple degrees of freedom for communication. In a  *n*_*T*_ by *n*_*R*_  channel, there are min{*n*_*T*_, *n*_*R*_} degrees of freedom. Spatial multiplexing gain (*r*) is associated with the system's transmission rate and demonstrates the way in which this rate gets increased with the increase in SNR. Spatial multiplexing gain cannot go over the total number of degrees of freedom. Therefore, the maximal multiplexing gain will be  min{*n*_*T*_, *n*_*R*_}. If *r* is known, we will get the data rate which is

*R*(SNR) ~ *r*_max_log_2_SNR bits/s/Hz.

The article "IoT-Oriented 6G Wireless Network System for Smart Cities" was published in 2022. Journal: Comput Intell Neurosci.

So, if data rate *R*  is known, we will get the multiplexing gain which is

(18) $$\begin{array}{c} r_{\text{max}}∼R|{\text{log}}_{2}\text{SNR}. \end{array}$$

The multiplexing gain and diversity of the proposed system are shown in Figure 5. From results, it has been found that the higher multiplexing gain and diversity can be achieved by using combined STBC-VBLAST.  Table 5 shows diversity and multiplexing gain.

## 3. Conclusion

Smart cities make better use of space, reduce traffic, provide cleaner air, and provide more efficient civic services, all of which improve people's quality of life. To enhance the services of smart city, an IoT-oriented 6G wireless network system will be very useful in processing vast amounts of incoming “sensory” data. An IoT-oriented relay assisted MIMO wireless network system for 6G is proposed and implemented in this work. The proposed system shows a significant performance on BER and capacity to overcome the key problems and challenges relating to wireless communication. Mathematical analysis and computer simulation are conducted to ensure the performance of the proposed system. It is found from BER performance that the developed scheme with relay does provide 1–17 dB gain with respect to direct connection. It is also found that this scheme provides 3 to 9 b/s/Hz improvement in performance of capacity at 5 to 10 dB by adding a different combination of STBC and VBLAST. Demonstration of the diversity and multiplexing gain proves that the proposed system is able to provide high data rates with reliable communication with interference for the IoT system. We are planning to develop massive antennas-based IoT system in future by increasing number of transmit and receive antennas with proposed encoding and decoding techniques.

## Figures and Tables

**Figure 1:** IoT-oriented 6G framework.

**Figure 2:** Communication layer for IoT-oriented MIMO wireless network.

**Figure 3:** BER performance of the proposed system.

**Figure 4:** Capacity of the proposed system.

**Figure 5:** Diversity and multiplexing gain.

**Table 1:** Encoding at source.

Antenna slot	I	II
1^st^	*x*_*k*,1,1,1_	*x*_*k*,2,1,2_
2^nd^	−*x*_*k*,2,2,1_^*∗*^	*x*_*k*,1,2,2_^*∗*^

**Table 2:** Re-encoding at relay for G21.

Antenna slot	-I-	-II-	-III-
1^st^	${\hat{x}}_{1}$	${\hat{x}}_{3}$	${\hat{x}}_{4}$
2^nd^	$-{\hat{x}}_{2}^{*}$	$-{\hat{x}}_{4}^{*}$	${\hat{x}}_{3}^{*}$

The article "IoT-Oriented 6G Wireless Network System for Smart Cities" was published in 2022. Journal: Comput Intell Neurosci.

**Table 3:** Re-encoding at relay for G211.

Antenna slot	-I-	-II-	-III-	-IV-
1^st^	${\hat{x}}_{1}$	${\hat{x}}_{3}$	${\hat{x}}_{5}$	${\hat{x}}_{6}$
2^nd^	$-{\hat{x}}_{2}^{*}$	$-{\hat{x}}_{4}^{*}$	$-{\hat{x}}_{6}^{*}$	${\hat{x}}_{5}^{*}$

**Table 4:** Re-encoding at relay for G2G211.

Antenna slot	-I-	-II-	-III-	-IV-	-V-	-VI-
1^st^	${\hat{x}}_{1}$	${\hat{x}}_{3}$	${\hat{x}}_{5}$	${\hat{x}}_{6}$	${\hat{x}}_{7}$	${\hat{x}}_{8}$
2^nd^	$-{\hat{x}}_{2}^{*}$	$-{\hat{x}}_{4}^{*}$	$-{\hat{x}}_{6}^{*}$	${\hat{x}}_{5}^{*}$	$-{\hat{x}}_{8}^{*}$	${\hat{x}}_{7}^{*}$

**Table 5:** Diversity and multiplexing gain.

	Diversity gain −Maximum (*d*_max_)	Spatial multiplexing gain- maximum (*r*_max_)
G2 (2 × 2)	4	1
G3 (3 × 3)	9	½
G4 (4 × 4)	16	½
H3 (3 × 3)	9	¾
H4 (4 × 4)	16	¾
VBLAST (2 × 2)	1	2
VBLAST (4 × 4)	1	4
VBLAST (4 × 4)	1	8
G21 (3 × 3)	3	2
G211 (4 × 4)	4	3
G2G211 (6 × 6)	6	4
G2G21111 (8 × 8)	8	6

## Data Availability

The data supporting the findings of this work are available within the article.
